# Evaluating Drug Risk Using GAN and SMOTE Based on CFDA's Spontaneous Reporting Data

**DOI:** 10.1155/2021/6033860

**Published:** 2021-08-27

**Authors:** Jianxiang Wei, Guanzhong Feng, Zhiqiang Lu, Pu Han, Yunxia Zhu, Weidong Huang

**Affiliations:** ^1^School of Management, Nanjing University of Posts and Telecommunications, Nanjing 210003, China; ^2^Key Research Base of Philosophy and Social Sciences in Jiangsu-Information Industry Integration Innovation and Emergency Management Research Center, Nanjing 210003, China; ^3^School of Internet of Things, Nanjing University of Posts and Telecommunications, Nanjing 210003, China

## Abstract

Adverse drug reactions (ADRs) pose health threats to humans. Therefore, the risk re-evaluation of post-marketing drugs has become an important part of the pharmacovigilance work of various countries. In China, drugs are mainly divided into three categories, from high-risk to low-risk drugs, namely, prescription drugs (Rx), over-the-counter drugs A (OTC-A), and over-the-counter drugs B (OTC-B). Until now, there has been a lack of automated evaluation methods for the three status switch of drugs. Based on China Food and Drug Administration's (CFDA) spontaneous reporting database (CSRD), we proposed a classification model to predict risk level of drugs by using feature enhancement based on Generative Adversarial Networks (GAN) and Synthetic Minority Over-Sampling Technique (SMOTE). A total of 985,960 spontaneous reports from 2011 to 2018 were selected from CSRD in Jiangsu Province as experimental data. After data preprocessing, a class-imbalance data set was obtained, which contained 887 Rx (accounting for 84.72%), 113 OTC-A (10.79%), and 47 OTC-B (4.49%). Taking drugs as the samples, ADRs as the features, and signal detection results obtained by proportional reporting ratio (PRR) method as the feature values, we constructed the original data matrix, where the last column represents the category label of each drug. Our proposed model expands the ADR data from both the sample space and the feature space. In terms of feature space, we use feature selection (FS) to screen ADR symptoms with higher importance scores. Then, we use GAN to generate artificial data, which are added to the feature space to achieve feature enhancement. In terms of sample space, we use SMOTE technology to expand the minority samples to balance three categories of drugs and minimize the classification deviation caused by the gap in the sample size. Finally, we use random forest (RF) algorithm to classify the feature-enhanced and balanced data set. The experimental results show that the accuracy of the proposed classification model reaches 98%. Our proposed model can well evaluate drug risk levels and provide automated methods for status switch of post-marketing drugs.

## 1. Introduction

Drug risk has always been a worldwide concern, and its most intuitive manifestation is adverse drug reactions (ADRs). The severity of adverse reactions of different drugs varies greatly. In some cases, it can even be fatal, which poses a great threat to people's health [1]. ADRs refer to harmful reactions of qualified drugs that have nothing to do with the purpose of medication under normal usage and dosage. Edwards and Aronson proposed a clearer definition of ADRs: “An appreciably harmful or unpleasant reaction, resulting from an intervention related to the use of a medicinal product, which predicts hazard from future administration and warrants prevention or specific treatment, or alteration of the dosage regimen, or withdrawal of the product [2].”

In order to reduce the harm caused by ADRs, the classification system of prescription (Rx) drugs and over-the-counter (OTC) drugs has become an internationally common model. According to the regulations of the US Food and Drug Administration (FDA), drugs are classified into Rx drugs and OTC drugs based on indicators such as toxicity and dependence [3]. Compared with Rx drugs, OTC drugs have less adverse reactions, and they can be purchased without a doctor's prescription to treat mild diseases. For OTC drugs, the China Food and Drug Administration (CFDA) further divides OTC drugs into two categories, namely, OTC-A drugs and OTC-B drugs, of which OTC-B is safer [4]. Therefore, drugs in China are divided into three categories, and the order of risk levels is Rx > OTC-A > OTC-B. At present, the drug regulatory authorities of many countries implement a re-evaluation system for post-marketing drugs, and switch Rx drugs and OTC drugs based on the frequency and severity of ADRs [5, 6]. As Brass argues, removal of the requirement for prescriptions saves both the health care professional and the patient time, but assessment of the ability of patients to use drugs in this manner is a critical component of the regulatory review [7]. This method mainly relies on the judgement of medical experts and lacks an automated risk identification technology. We hope to build a multi-classifier to determine whether a drug belongs to one of the above three categories by evaluating ADRs, in order to provide an objective and automatic method for the status switch of drugs. Furthermore, the accurate classification of drugs will provide more convenience for patients' medication, while reducing the risk of ADRs as much as possible.

The ADR reports used in this experiment all originate from CFDA's spontaneous reporting system (SRS). Spontaneous reporting means that medical workers voluntarily report suspicious ADRs discovered in the clinic to drug manufacturers, adverse reaction monitoring agencies, drug regulatory departments, etc. [8]. SRS is suitable for wide deployment in various regions and can collect large amounts of ADR data [9]. Nowadays, most members of WHO Uppsala Monitoring Centre (UMC) have adopted this system [10]. However, the information in many reports is too rough, which may affect the causality of adverse reactions, leading to over or under attribution [11]. At the same time, incomplete or missing reports make it impossible to calculate the incidence of ADR accurately. Therefore, it is necessary to standardize the original data and use the method of signal detection to extract effective information. At present, the commonly used signal detection method for ADRs is disproportionality analysis (DPA) [12, 13]. The proportional reporting ratio (PRR) used in this paper is one of the DPA methods. Based on the PRR method, we can build a data matrix with drugs as samples, ADR symptoms as features, and signal detection results as feature values. The last column of the matrix represents the category label of each drug.

Since the overall data contains many types of ADRs, and only part of the adverse reactions is caused by one drug, this data matrix is high-dimensional and sparse. A large number of features can increase interference noise and may obscure some important ADR data. In order to improve the classification accuracy, it is necessary to perform feature selection on the data set. The principle of feature selection is to use detection methods to evaluate all features from the data set, and retain features that are efficient and reliable for data classification [14]. The experiment uses machine-learning methods to extract features with high importance scores.

Considering that the high-dimensional feature space contains a lot of information about ADR symptoms, we cannot simply keep important features and delete those that are not helpful for classification, because this method may cause some serious ADR features to disappear, making it difficult to accurately evaluate the potential risks of drugs. On the basis of retaining the existing ADR features, we hope to expand the feature space with more effective data that are helpful for the classification. Goodfellow et al. proposed the concept of generative adversarial networks (GANs) in 2014 [15]. As a popular theory in deep learning in recent years, GAN has achieved outstanding performance in data generation. Therefore, according to the feature selection data, we use GAN to generate similar artificial data, which are added to the feature space to achieve feature enhancement.

In terms of sample space, the number of Rx drugs and OTC drugs in our ADR data set is extremely imbalanced. Traditional classification techniques perform poorly on this type of data because they tend to favor the majority class. The synthetic minority over-sampling technique (SMOTE) algorithm proposed by Chawla et al. is one of the most representative external methods to balance data sets through resampling [16]. We use SMOTE to balance the data set by adding samples based on k-nearest neighbors in the minority class. The samples of Rx, OTC-A, and OTC-B drugs will reach a balanced state after SMOTE resampling, which lays a data foundation for using conventional random forest (RF) classification algorithm.

The purpose of this paper was to build a high-accuracy drug risk level classification model, which can be deployed in the Chinese spontaneous reporting system. When a drug manufacturer applies to the drug regulatory authority for drug category switch, CFDA organizes medical experts to conduct drug risk assessment. In this process, the proposed model can automatically identify the drug category according to the ADR monitoring data after the drug is put on the market, which can provide auxiliary decision support for experts.

## 2. Related Work

With the development of computer science, the use of machine learning to solve ADR problems is common and widely used, which makes great contribution to the control of medication risks. In 2011, Pouliot et al. used more than 480,000 molecular activity data in the PubChem database to establish a logistic regression model to predict the level of ADRs that may be caused by target drugs [17]. The results show that 75% of the adverse reaction signals mined by this model could be verified by relevant medical literature or drug instructions. In the same year, Santiago et al. proposed a new ADR detection method, which compared and screened the drugs involved in the adverse reaction signals, and then obtained the final mining results [18]. In this way, the sensitivity of mining adverse reactions related to rhabdomyolysis reached 70%, and the positive detection rate reached 45%. In 2013, Chen et al. realized the identification of high-risk proteins and the discovery of potential adverse reaction mechanisms through the analysis of the high-risk protein network of ADRs [19]. This study analyzed the data of drug target proteins, protein pathways, and proteins related to adverse reactions. The results found a total of 41 ADR protein subnetworks, and found that certain biological enzymes and transport proteins are the key factors causing adverse reactions.

In the field of risk mining of ADRs, researchers have conducted a lot of research on various types of spontaneous report databases and have achieved sufficient results. In 2014, Roberto et al. used signal detection methods to conduct data mining, trying to detect the serious cardiovascular adverse reaction signals of triptans drugs [20]. The results show that triptans drugs are related to a variety of adverse reactions such as ischemic cerebrovascular complications. In 2015, Mai et al. conducted data mining in the spontaneous report database and found that the use of statin drugs may increase the risk of rectal cancer or pancreatic cancer [21]. In 2018, Scholl et al. proposed a prediction-model-based approach to improve the efficiency of full database screening [22]. The AUC value and the ratio of potential signals of this method have been greatly improved compared with traditional signal detection methods. In 2019, to resolve entity-level ADR classification tasks, Alimova and Tutubalina investigated deep neural network models in the natural language processing (NLP) field based on various ADR corpus [23].

In recent years, researchers have analyzed ADR from multiple perspectives such as patient age and drug interaction, and have proposed many new risk detection methods. In 2020, Martocchia et al. evaluated the incidence of adverse events and drug-drug interactions exposed to polypharmacy and proposed that the application of certain software programs could significantly reduce the incidence of adverse events at every level of healthcare [24]. In 2021, Giangreco and Tatonetti pointed out that detection of ADR is challenging due to dynamic biological processes during ontogeny, which alter pharmacokinetics and pharmacodynamics [25]. The population modeling technique they proposed exhibited normally distributed and robust ADR risk estimation at all development stages of children. In the same year, Mehta et al. reviewed the risk assessment methods of prescription drug and developed more than two dozen prescription drug-based risk indices, which differ significantly in design, performance, and application [26].

Regarding China's spontaneous report data, scholars have integrated and evaluated ADR information, and have begun to measure drug risks in an intelligent way. In 2015, Ge et al. used the NLP method to extract knowledge of adverse reactions in a large number of Chinese clinical narrative texts [27]. Based on the results of knowledge extraction, they established a knowledge base corresponding to drugs and adverse reactions, and set up a website to provide online query and to download ADR information. In 2020, we compared four drug-risk prediction models using machine-learning methods as classifiers, and determined the best risk prediction framework [28], with a classification accuracy rate of 95%.

In order to further improve the classification accuracy so that the risk prediction model can be applied in practice, this paper is based on the previous research, and realizes the feature enhancement of high-dimensional ADR feature space through the combination of GAN and feature selection. Furthermore, by comparing with our previous models, we propose a better predictive model for evaluating drug risks.

## 3. Materials

ADR reports used in this study were obtained from the CFDA in Jiangsu Province. The data set covered a total of 985,960 ADR reports in Jiangsu Province from 2011 to 2018, including report ID, report address, patient age, gender, drug name, and ADRs symptom. Due to invalid and duplicate reports, we deleted data with no reference value and standardized the names of drugs and ADR symptoms. Then 1,047 drug names and 751 ADR symptoms were prepared. In more detail, for each drug, the ADR mentioned in one report would increase the total of corresponding ADR symptoms by one. The result of the final statistics is a table with the drug names corresponding to the frequency of all types of ADRs. Data set could be described as the following.

Sample space:

(1) $$\begin{array}{c} X=\left\{x_{1},x_{2},\ldots ,x_{m}\right\}. \end{array}$$

Here, *m* = 1047. The drugs and ADRs make up the sample space together. Drugs are the samples and ADRs are the features.

Feature vector:

(2) $$\begin{array}{c} x_{i}=\left(x_{i1},x_{i2},\ldots ,x_{i\;d}\right)\in X. \end{array}$$

Here, *d* = 751. Every sample is composed of *d* features, and *x*_*i*_ is one of the feature vectors in sample space, where *x*_*i*  *d*_ represents the frequency under the matching drug-ADR pairs.

According to the China Medical Information Platform, we manually labeled all drug samples, with values 0, 1, and 2 representing Rx, OTC-A, and OTC-B, respectively.

The statistical results in Table 1 show that Rx drugs account for a high proportion, while the two categories of OTC drugs are the opposite, which means that the classes in the data set are imbalanced.

## 4. Methods

### 4.1. Model Framework

Figure 1 shows the flowchart of the proposed model. The model is mainly divided into four stages: signal detection stage, feature enhancement stage, minority expansion stage, and RF classification stage.

1. Signal detection stage: the first step of the proposed model is to use signal detection on the preprocessed spontaneous report data, and calculate the PRR value of the drug-ADR pairs to obtain the ADR imbalanced data set.
2. Feature enhancement stage: based on the ADR imbalanced data set, the model selects the top 200 features of classification importance, and uses GAN to generate artificial features that meet the real data distribution. The generated features are added to the imbalanced ADR data set, so that the feature space contains more effective features, which can improve the classification accuracy. So far, the feature-enhanced ADR imbalance data set has been obtained.
3. Minority expansion stage: SMOTE is used to expand the minority samples (OTC-A and OTC-B) to equalize the number of the three categories of drugs, which helps to obtain a feature-enhanced ADR balanced data set.
4. RF classification stage: the RF algorithm is used to classify the feature-enhanced ADR balanced data set. Finally, we analyze the results of the proposed model based on multiple indicators, and further evaluate the risks of postmarketing drugs.

### 4.2. Signal Detection

The DPA method is currently the most used ADR signal detection technology [29]. DPA is used to measure the disproportion or imbalance of the sample distribution in the database. If the number of occurrences associated with drug and adverse event is greater than the expected number or the number of other combinations, it is considered that there is a potential connection between the drug and the adverse event, which may be a positive ADR signal. Calculation of DPA is based on the principles using the two-by-two contingency table.

Proportional reporting ratio (PRR) is one of the DPA methods, which was proposed in 2001 by Evans of the British Medical Regulatory Authority [30], and it is a key method for ADR signal detection in the world. The calculation of PRR is similar to the relative risk in epidemiological studies, which is used to quantify the strength of the drug-ADR association. According to Table 2, the formula to compute PRR value is

(3) $$\begin{array}{c} \text{PRR}=\frac{\left(A/\left(A+B\right)\right)}{\left(C/\left(C+D\right)\right)}. \end{array}$$

Formula (3) indicates that if the PRR value of a drug-ADR pair is larger, the relative risk is higher, so the risk of the adverse reaction corresponding to the drug is greater. In our study, after calculating the PRR value of all drug-ADR pairs based on statistical data, the data matrix is established with drugs as the sample, ADR as the feature, and PRR results as the matrix value. The last column of the data matrix is the category label of each drug, where Rx is “0,” OTC-A is “1,” and OTC-B is “2.” Due to the quantitative difference among the three categories of drugs, we got the ADR imbalance data set.

### 4.3. Feature Enhancement

Since the overall data contain many types of ADRs, and only part of the adverse reactions is caused by one drug, this data matrix obtained by PRR is high-dimensional and sparse. In order to improve the model's classification accuracy of this data set, we expand the effective ADR data in the feature space to achieve feature enhancement.4.3.1. Algorithm ID4 is Used for Feature Selection (FS)

In the process of decision tree attribute splitting, the Gini index is used to calculate the contribution of a single feature for the correct classification. During tree growth, the purity measure of split at node *k* is:

(4) $$\begin{array}{c} \text{Gini}\left(p_{k}\right)=\overset{n}{\underset{k=1}{\sum }}p_{k}\left(1-p_{k}\right)=1-\overset{n}{\underset{k=1}{\sum }}p_{k}^{2}. \end{array}$$

In formula (4), *p*_*k*_ represents the probability that the sample is correctly classified at node *k*. The sample is divided into different branches to produce their branch sets  *T*^*v*^, and the purity measure is as follows:

(5) $$\begin{array}{c} {\text{Gini}}_{\text{index}\left(T,k\right)}=\overset{V}{\underset{v=1}{\sum }}\frac{\left|T^{v}\right|}{\left|T\right|}\text{Gini}\left(T^{v}\right). \end{array}$$

*T* represents the current divided set, and the Gini index reflects the probability that any two branch sets are inconsistent. A smaller Gini index in formula (5) indicates that the branch set is purer, which also means that the classification accuracy will be higher. Therefore, node *k* strives to meet the minimum purity:

(6) $$\begin{array}{c} k^{*}=\arg\underset{k}{\min}{\text{Gini}}_{\text{index}\left(T,k\right)}. \end{array}$$

The feature *f*_*i*_ is the classification basis of node *k*, and left and right branches can be obtained. They are measured according to the Gini changes of the branches:

(7) $$\begin{array}{c} {\text{Gini}}_{\left(f_{i},k\right)}=\text{Gini}\left(P_{k}\right)-\text{Gini}\left(P_{1}\right)-\text{Gini}\left(P_{r}\right). \end{array}$$

Gini(*P*_1_), Gini(*P*_*r*_) represent the Gini index of the left and right branches, respectively. After calculating Gini_(*f*_*i*_, *k*)_ in formula (7), the importance of the feature *f*_*i*_ in the *j*-th tree is:

(8) ImjGini=∑m∈MGinifi,k.

The importance of feature *f*_*i*_ on a single tree is calculated by formula (8). Furthermore, in the total number of *m* trees, the feature *f*_*i*_ appears when part of the tree nodes split. Then, the overall importance of measuring feature *f*_*i*_ is:

(9) Imfi=∑j=1mImjGini.

In order to select features that are more effective for classification, the features are ranked in the descending order of importance calculated by formula (9). The first 200 main features are retained as the basis for the next step of GAN feature generation.

#### 4.3.1. Use GAN to Generate New Features

GAN is a generative model based on zero-sum game theory. It includes a generative model (*G*) and a discriminant model (*D*), both of which are based on neural networks. In the training process of *G* and *D*, *G* generates data similar to the true value through the noise space *z*. The goal of *D* is to distinguish between real data or generated data. Generator and discriminator are iteratively optimized with each other, so that their performance continues to improve. In the end, the two models reached a Nash equilibrium. At this time, the data generated by GAN approximates the real data [31, 32]. The evaluation formula of GAN is as follows:

(10) $$\begin{array}{c} \underset{G}{\min}\underset{D}{\max}V\left(D,G\right)=E_{x∼P_{\text{data}}\left(x\right)}\left[\log\;D\left(x\right)\right]+E_{z∼P_{z}\left(z\right)}\left[\log\left(1-D\left(G\left(x\right)\right)\right)\right]. \end{array}$$

In formula (10), *x* is the real data, which conforms to the *P*_data_(*x*) distribution; *z* is the hidden space noise, which conforms to the *P*_*z*_(*z*) distribution. *V*(*D*, *G*) represents the degree of difference between the real sample and the generated sample. Formula (10) indicates that when the discriminator maximizes the difference and the generator minimizes the difference between the real samples and the generated samples, after multiple rounds of iterative training, realistic data can be obtained.

We use two sets of neural networks to construct *G* and *D*, respectively. The key factors in the training process are gradient descent, alternate training, and back propagation. The training steps in the experiment are summarized as follows:

Step1: select some samples {*z*_1_, *z*_2_,…, *z*_*m*_} from the input random noise *P*_*z*_(*z*).
Step2: sampling from the original training set, the number of samples {*x*_1_, *x*_2_,…, *x*_*m*_} is the same as the noise samples.
Step3: set the parameter of *D* to *θ*_*d*_, and use the gradient ascent algorithm in formula (11) to update the discriminator:
  (11) $$\begin{array}{c} \nabla \frac{1}{m}\overset{m}{\underset{i=1}{\sum }}\left[\log\;D\left(x_{i}\right)+\log\left(1-D\left(G\left(z_{i}\right)\right)\right)\right]. \end{array}$$
Step4: repeat steps 1–3 for *k* times, and then update *G* once.
Step5: set the parameter of *G* to *θ*_*g*_, and use the gradient descent algorithm in formula (12) to update the generator:
  (12) $$\begin{array}{c} \nabla \frac{1}{m}\overset{m}{\underset{i=1}{\sum }}\log\left(1-D\left(G\left(z_{i}\right)\right)\right). \end{array}$$
Step6: repeat steps 1–5 until the GAN model converges.

Input the features selected in Step 4.3 (1) into GAN to generate an equal number of artificial ADR features. These generated features satisfy the real value distribution and are consistent with the original data. Use generated ADR features as real data to expand the feature space in order to enhance the risk characteristics of the drugs. Now, we obtain a feature-enhanced ADR imbalance data set.

### 4.4. Synthetic Minority Over-Sampling Technique (SMOTE)

After adding the generated ADR features to the data set, the number of effective features in the sample is increased, which is helpful for subsequent classification. However, the proportions of Rx, OTC-A, and OTC-B drugs in the data set are quite imbalanced. Traditional classification algorithms will seriously bias the majority class and ignore the minority class, leading to deviations in the result. Therefore, for the imbalanced data set in this experiment, we use the SMOTE algorithm to expand the minority samples before classification.

The core of SMOTE is to insert randomly generated new samples between the minority samples and their neighbor samples [33]. This can increase the number of minority samples and improve the class imbalance distribution of the data set [34]. The steps of the SMOTE are as follows:

Step 1: the number of majority samples in the data set is *N*^+^, and the number of minority samples is *N*^−^. Calculate the imbalance ratio IR and oversampling rate *K* of the original data set:
  (13) $$\begin{array}{c} \text{IR}=\frac{N^{+}}{N^{-}}. \end{array}$$
Round down IR in formula (13) to get the oversampling rate *K*:
  (14) $$\begin{array}{c} K=\left\lfloor \text{IR}\right\rfloor , \end{array}$$
(⌊.⌋ means rounding down the data.)
Step 2: for each minority sample  *x*_*i*_, calculate the Euclidean distance with other minority samples, and find the *k* nearest neighbors. The Euclidean distance is calculated as follows:
  (15) $$\begin{array}{c} d\left(x_{i},x_{j}\right)=\sqrt{\left(x_{i1}-x_{j1}\right)+\left(x_{i1}-x_{j2}\right)+\cdots +\left(x_{ip}-x_{jp}\right)}. \end{array}$$
Step 3: according to the oversampling rate *K* in formula (14) and Euclidean distance *d*(*x*_*i*_, *x*_*j*_) in formula (15), K samples are randomly selected from the *k* nearest neighbors with replacement, and mark them as $\;\bar{x_{i}}\left(i=1,2,\ldots ,K\right)$. Calculate the difference between *x* and $\bar{x_{i}}$ as $\left(x-\bar{x_{i}}\right)$.
Step 4: use formula (16) to synthesize each new sample *x*_new_^*i*^:
  (16) $$\begin{array}{c} x_{\text{new}}^{i}=x+\text{rand}\left(0,1\right)\times \left(x-\bar{x_{i}}\right),\;i=1,2,\ldots ,K, \end{array}$$
(rand(0,1) returns a random value in the interval (0,1).)
Step 5: repeat the above steps to synthesize *K* · *N*^−^ data artificially for the minority samples.

After the above steps, the three categories of Rx, OTC-A, and OTC-B in the data set have reached the same number, which improves the data distribution in the sample space. As a result, we obtained the feature-enhanced ADR balanced data set, which laid a data foundation for classification.

### 4.5. Random Forest Classifier

We use the random forest (RF) algorithm to classify the feature-enhanced ADR balanced data set. The RF algorithm is a machine-learning method proposed by Breiman in 2001 [35]. Its main idea is to build a forest containing multiple decision trees. Each decision tree adopts a random decision-making method in this process and remains independent during classification. Each decision tree in the RF will predict the outcome. Finally, all the outcomes are integrated by voting, and the class with the highest probability is selected as the classification result [36]. The steps of RF classification are as follows:

  Step 1: assume that the number of samples in the training set (*S*) is *N*. We randomly select *N* samples from the training set with replacement as the training set *S*_*i*_ of the decision tree *T*_*i*_. A total of *K* training sets are extracted to construct *K* decision trees.
  Step 2: the dimension of the features in each sample is *M*. In the process of training the decision tree, *m* subsets are randomly selected from all the features of each node.
  Step 3: the decision tree selects a node with the best splitting ability in the feature subset to split.
  Step 4: each decision tree grows to the maximum extent and does not require pruning.
  Step 5: all decision trees constitute the final RF, and the result of the classification is determined by voting.

### 4.6. Evaluation Metrics

Traditional classification algorithms use precision metric to determine the performance of the classifier on the data set. Although it is effective for balanced data, there will be obvious deviations for unbalanced data.

For example, for tumor detection data, the proportion of benign is very high, and the proportion of malignant is very low. High accuracy can be obtained by classifying all tumors as benign. However, this classification is meaningless, because for issues such as disease detection, disaster prediction, and credit fraud, the minority samples are of great significance and need to be focused on.

For a given sample set, we can get the confusion matrix by comparing the real class with the class predicted by the classifier [37]. As shown in Table 3, there are four situations:

According to the confusion matrix in Table 3, the following evaluation metrics can be calculated:

(1) Precision: Tthe precision rate reflects the proportion of true positive samples in the positive class judged by the classifier.
  (17) $$\begin{array}{c} \text{Precision}=\frac{\text{TP}}{\text{TP}+\text{FP}}. \end{array}$$
(2) Recall: the recall rate reflects the proportion of positive classes that are correctly classified in the total positive classes.
  (18) $$\begin{array}{c} \text{Recall}=\frac{\text{TP}}{\text{TP}+\text{FN}}\text{.} \end{array}$$
(3) Accuracy: the accuracy rate reflects the classifier's ability to predict the positive and negative classes correctly.
  (19) $$\begin{array}{c} \text{Accurary}=\frac{\text{TP}+\text{TN}}{\text{TP}+\text{FN}+\text{FP}+\text{TN}}\text{.} \end{array}$$
(4) *F*-measure: F1 is the harmonic mean of precision and recall [38], and is a commonly used evaluation criterion for classification of imbalanced data sets. After obtaining Precision and Recall in formulas (17) and (18), F1 can be calculated as
  (20) $$\begin{array}{c} \text{F}1=\frac{\left(1+\beta^{2}\right)*\text{Recall}*\text{Precision}}{\beta^{2}*\text{Recall}+\text{Precision}}, \end{array}$$
*β* is the scale factor, and its usual value is 1.
(5) Macro-avg: macro average is a commonly used evaluation index for multi-classification problems, which can measure the overall situation of the classifier [39]. For formulas (17), (18), and (20), the values of each class are first calculated, and then the average values of all the classes are calculated.
  (21) $$\begin{array}{c} {\text{Macro}}_{P}=\frac{1}{n}\overset{n}{\underset{i=1}{\sum }}P_{i}. \end{array}$$
  (22) $$\begin{array}{c} {\text{Macro}}_{R}=\frac{1}{n}\overset{n}{\underset{i=1}{\sum }}R_{i}. \end{array}$$
  (23) $$\begin{array}{c} {\text{Macro}}_{\text{F}1}=\frac{2*{\text{Macro}}_{P}*{\text{Macro}}_{R}}{{\text{Macro}}_{P}+{\text{Macro}}_{R}}, \end{array}$$
*n* represents the number of classes, *i* represents each class.
Macro average in formula (21)–(23) treats each class equally, and its results are more susceptible to minority samples. In other words, macro average has advantages in highlighting the classification performance of minority samples.
(6) Weighted-avg: The weighted average can comprehensively evaluate the accuracy of classification [40]. By assigning weight to each class, the average value of all classes is calculated according to Precision, Recall, and F1 in formulas (17), (18), and (20).
  (24) $$\begin{array}{c} {\text{Weighted}}_{P}=\overset{n}{\underset{i=1}{\sum }}\frac{C_{i}}{\left|C\right|}*P_{i},\\ {\text{Weighted}}_{R}=\overset{n}{\underset{i=1}{\sum }}\frac{C_{i}}{\left|C\right|}*R_{i},\\ {\text{Weighted}}_{\text{F}1}=\overset{n}{\underset{i=1}{\sum }}\frac{C_{i}}{\left|C\right|}*{\text{F}1}_{i}, \end{array}$$
 *n* represents the number of classes, *i* represents each class, |*C*| represents all samples, and *C*_*i*_ represents the samples included in one class.
(7) Receiver Operating Characteristic (ROC) Curve
Among the evaluation criteria for imbalanced data sets, the ROC curve is a generally accepted and comprehensive evaluation criterion [41]. The ROC curve has a false positive rate (FPR=FP/(FP+TN)) on the horizontal axis and a true positive rate (TPR=TP/(TP+FN)) on the vertical axis. Through the cross-validation method, multiple sets of point pairs (FPR, TPR) of the classifier can be obtained. Then, draw them to a plane and connect them to form the final ROC curve. The ROC curve is a very intuitive way to evaluate the classifier. The closer the curve is to the upper left corner, the better the performance of the classifier.
Area under curve (AUC) refers to the area enclosed by the ROC curve and the coordinate axis. The value of this area will not be greater than 1. Since the ROC curve is generally above the line *y*=*x*, the value of AUC ranges between [0.5, 1]. The closer the AUC is to 1, the higher the accuracy of classification.

### 4.7. Experiment Design

In order to observe the effect of the abovementioned methods on the classification of CFDA's spontaneous reporting data, this paper designs three comparative models.

In the first model (*Model 1. RF*), we use the data set after PRR signal detection as the basis (ADR imbalance data set). The total number of three categories of drugs is 1047, including 887 Rx drugs (label = 0), 113 OTC-A drugs (label = 1), and 47 OTC-B drugs (label = 2). The data space contains 751 features (ADRs). Use traditional RF algorithm for classification.

In the second model (*Model 2. SMOTE* *+* *RF*), we use the SMOTE algorithm to expand the data set after PRR signal detection, so that the quantity of each category reaches a balance (ADR balanced data set). The total number of drugs is 2661, and the number of Rx (label = 0), OTC-A (label = 1), OTC-B (label = 2) drugs are equal, all of which are 887. The data space contains 751 features. Then, use RF for classification.

In the third model (*Model 3. FS_GAN* *+* *SMOTE* *+* *RF*), we will use the model proposed in this paper. The ADR data set used by this model has also been improved in terms of samples and features (feature-enhanced ADR balanced data set). The total number of drugs is 2661, and the number of Rx (label = 0), OTC-A (label = 1), and OTC-B (label = 2) drugs are equal, all of which are 887. The data space contains 951 features (751 original + 200 generated). Finally, the RF algorithm is used for classification.

The experiment in this article consists of two sections. In the first section, the above three models all use 70% of the sample space as the training set, and the remaining 30% as the test set. Then, we observe the classification results based on the test set. In the second section, we input the actual ADR data collected by CFDA into all three trained models and observe the results. Furthermore, it means that the three models use the same actual ADR data after PRR (1047 samples) as the test set.

## 5. Results

### 5.1. Results of the Classifiers Using the Test Set

In this section, the three models use 70% of their sample space for training, and use the remaining 30% as the test set. The sample size in the test set of each model is calculated as follows:

  Sample size (model 1) = 1047 × 30% = 315
  Sample size (model 2) = 2661 × 30% = 799
  Sample size (model 3) = 2661 × 30% = 799

Therefore, the sample size of test sets used by each model is 315 (Model 1), 799 (Model 2), and 799 (Model 3). The confusion matrices obtained by classification are shown in Figure 2:

Figure 2 shows three confusion matrices of three models, from which it can be seen that Model 3 (FS_GAN + SMOTE + RF) has the largest proportion of results on the diagonal, which means it has the highest accuracy of classification. More detailed evaluation indicators are shown in Table 4.

Table 4 shows the evaluation metrics of the three models based on their test set. Model 1 is biased towards the majority class, so the prediction results for OTC-A (label = 1) and OTC-B (label = 2) are very poor, and its accuracy is the lowest, only 84.44%. Model 2 balances the data set and can predict most of the OTC drugs (label = 1, 2), with an accuracy rate of 91.99%. Model 3 has the highest prediction accuracy for minority samples, reaching 96.25%. From the macro average and weighted average metrics, Model 1 is the worst, Model 2 ranks second, and Model 3 has the best performance.

### 5.2. Validation Results Based on Actual ADR Data

In the verification section, the actual ADR data are used as the test set to validate the prediction results of the three trained models in Section5.1. The test sample size of the three models equals to that of the actual ADR data, which is 1047.

The confusion matrices corresponding to the three models are shown in Figure 3.

Figure 3 illustrates the confusion matrices of the three models using the actual ADR data after PRR signal detection as the input (sample size_1,2,3_=1047). In the confusion matrix, the blocks on the diagonal indicate the number of correctly classified labels. For each model, the sum of correctly predicted data is calculated as follows:

  Sum (Model 1) = 874 + 41 + 13 = 928
  Sum (Model 2) = 845 + 102 + 44 = 991
  Sum (Model 3) = 876 + 105 + 44 = 1025

Under the verification of the same data set, the number of samples correctly predicted by Model 3 is the largest, reaching 1025, which is higher than 928 of Model 1 and 991 of Model 2. This result means that Model 3 has the highest prediction accuracy. More detailed evaluation metrics are shown in Table 5.

Table 5 shows the evaluation metrics of the three models using the same actual ADR data. Among them, the accuracy of Model 1 is the lowest, only 88.63%. Model 2 has significantly improved its ability to recognize minority classes, with an accuracy rate of 94.65%. The results indicate that Model 3, which uses the combination of feature enhancement (FS_GAN) and SMOTE, has a higher accuracy than Model 2, which only uses SMOTE, reaching 97.90%. The other metrics such as macro average and weighted average also indicate that the performance of Model 3 is the best.

Figure 4 shows the ROC curves and AUC values of the three models. It indicates that Model 1 using only the RF algorithm has the worst classification result for the imbalanced ADR data set, and its AUC value of 0.85 is also the lowest. For the latter two models after SMOTE, the ROC curve of Model 3 with feature enhancement (FS_GAN) is closer to the (0,  1) point. The AUC value of Model 3 is also the highest among them, reaching 0.99.

## 6. Discussion

The classification results on CFDA's actual ADR data show that the accuracy of Model 1 reaches 88.63%, which seems to be a good result. However, by observing the index of the recall rate of Model 1, we can find that the recall rate of label 1 is 0.36, and the recall rate of label 2 is 0.28. In other words, Model 1 predicts most of the samples as the majority class (label = 0), so it obtains high accuracy. As mentioned in Part 4, such classification is meaningless, because the minority classes are not identified. The latter two models use SMOTE to expand the minority samples, and the number of Rx (label 0), OTC-A (label = 1), and OTC-B (label = 2) drugs reached a balance. Therefore, the recall rate and F1 index are both very high, which indicates that they have a good classification effect on the three categories of drugs.

By comparing the three models, we found that Model 3 is the best, with an accuracy of 97.90%. The Precision, Recall, and F1 index corresponding to the three categories of labels in Model 3 are all higher than Model 2. Especially, for the recognition of minority classes (label = 1 and label = 2), their prediction success rates in Model 3 have been greatly improved.

From the perspective of macro averaging, Model 3 has achieved excellent performance. The macro average takes the arithmetic average of all classes, which means that each class is treated equally during classification, so that the impact of small samples on the results can be more clearly highlighted. The macro-average value of Model 3 is higher than Model 1 and Model 2, so Model 3 is more suitable for the classification of imbalanced samples.

Compared with the macroaverage, the weighted average is more inclined to be affected by the majority class, because the majority category accounts for a larger proportion of the entire samples, and the corresponding weight is also larger. The weighted average of each metric of Model 3 is 0.98, which is the highest among all classifiers.

From the perspective of the ROC curve, the ROC curve of Model 3 is closest to the (0,  1) point among the three, which indicates that Model 3 has the highest classification accuracy rate for imbalanced data sets. This result is confirmed again from the perspective of AUC. The AUC value of Model 3 is 0.99, which is higher than 0.85 of Model 1 and 0.97 of Model 2.

Based on the same CFDA's ADR data, we compared the model proposed in this paper (Model 3) with the model established by our previous work in multiple evaluation indicators. Previously, we compared the prediction results of four machine-learning algorithms, including RF, gradient boost (GB), logistic regression (LR), and AdaBoost (ADA), in the steps of PRR signal detection and SMOTE oversampling, and finally obtained the optimal combination PRR-SMOTE-RF. Through the comparison of experimental results, the accuracy of Model 3 proposed in this paper is 0.98, which is higher than the 0.95 of the previous model PRR-SMOTE-RF. This comparison shows that for ADR samples with obscure features, Model 3 will achieve better prediction results. From the perspective of ROC curves, Model 3 in this paper also has better performance. The AUC value of Model 3 reached 0.99, higher than the 0.97 of PRR-SMOTE-RF, which means that Model 3 has better classification performance for imbalanced data sets. Finally, we can determine that the model with feature enhancement proposed in this paper has better performance on actual ADR data, and has a higher accuracy rate for drug risk prediction.

For the high-dimensional ADR feature space, it is difficult for us to remove redundant features to improve the classification accuracy. The reasons mainly include the following two points. On the one hand, the feature space contains the adverse reactions corresponding to the drugs. If a part of the features that have no effect on the classification are deleted, the potential risks of some drugs may be ignored, leading to deviations in the classification of drugs. For drugs with serious adverse reactions, ignoring their ADR features is fatal, which will cause great harm to patients in the future. On the other hand, additional experiments prove that deleting some redundant features does not improve the classification accuracy very well. We hope to add some effective data that are helpful for classification in the feature space to achieve feature enhancement. In addition, GAN has great advantages in data generation. Through multiple training iterations, GAN can learn about the potential data distribution in the samples and generate similar artificial data. Therefore, when the number of samples is sufficient, GAN-based feature enhancement is an efficient method to solve such problems.

The experimental results prove that it is effective to use feature enhancement technology and minority oversampling at the same time for high-dimensional imbalanced data sets. Compared with the previous PRR-SMOTE-RF framework that does not use feature enhancement, the model proposed in this paper has a higher classification accuracy on the same ADR data set. Other evaluation indicators also confirmed this conclusion. Furthermore, the results indicate that it is effective to use GAN to generate artificial data to improve the overall data distribution in the feature space. In other words, on the basis of minority oversampling of imbalanced data sets, feature enhancement can help achieve more accurate classification. At the same time, this method retains all existing ADR features, thus avoiding the risk evaluation deviation caused by lack of features.

Furthermore, we compare the artificial data generated by GAN with the real data in the ADR data set. Since the data set contains a variety of ADR symptoms, and a drug causes only a small part of the adverse reactions, the data matrix after PRR signal detection is high-dimensional and sparse. The proportion of nonzero elements in the original ADR imbalanced data set is 1.73%. For the top 200 features screened by FS, the proportion of nonzero elements is 5.02%; while for the artificial data generated by GAN, its proportion is 4.85%. This result indicates that artificial data and real data have a high degree of similarity in numerical form. The artificial features generated by GAN satisfy the spatial distribution characteristics of the original data. More specifically, the data distribution of artificial data and real data is similar. Therefore, adding artificial features to the ADR imbalanced data set can improve the sparsity of its feature space. This once again verified that it is feasible to use GAN to achieve feature enhancement.

Through the above analysis, we can draw conclusion that Model 3 (FS_GAN + SMOTE + RF) is more suitable for the prediction of CFDA's spontaneous report data. When choosing this model to evaluate drug risks, we need to conduct further analysis on misclassified drugs. On the one hand, the proposed model has deviation, which can make some medicines misclassified. On the other hand, the adverse reaction corresponding to the drug does not match the class it belongs to, which leads to the wrong classification. In view of the above two situations, experts will reevaluate the misclassified drugs. For drugs that do not match their category, they need to switch among Rx, OTC-A, and OTC-B to control the risks of drugs.

However, this study has several limitations including the following:

1. Sample size: the research used 985,960 spontaneous reports from 2011 to 2018 provided by CFDA in Jiangsu Province as experimental data, which can visually verify the effectiveness of the proposed model. However, it is difficult to verify the model's evaluation results of drug risks on a larger scale because the sample size is not sufficient. Since Chinese spontaneous report database is not open to the public, we cannot further obtain more updated samples. This results in the limited availability of relevant data due in part to the high cost of collection of such specialized data. During the preprocessing stage, we deleted a large amount of incomplete and worthless ADR data, which led to a reduction in the sample size. At the same time, the time span and the quality of the SRS are also key factors affecting sample size.
2. Feature enhancement: in the process of feature selection, we use the relative importance score to rank the ADR features. This selection method may cause some features that have an important impact on the classification to be ranked lower, or even be obscured. We discussed the characteristics of artificial data and real data above, and proved the similarity between the two in terms of data distribution. However, how to further measure the difference between artificial data and real data requires in-depth research in the follow-up work.
3. Drug interaction: in this study, aspects such as adverse reactions caused by drug interactions are not investigated as these factors are beyond the scope of this research. Potentially, the analysis of ADRs caused by the interaction of different drugs involved in the collected spontaneous reports will help us understand the process of adverse reactions and further clarify the risks of drugs.

In summary, the results of this study indicate that it is feasible to use GAN and SMOTE to classify imbalanced ADR data from CFDA's spontaneous reporting database. This classification can help us understand the applicable population of drugs. Through the evaluation of the classification results, we can further identify the drug risks faced by consumers in a variety of situations, so as to reduce the occurrence of unexpected problems. At the same time, the evaluation of drug risks may help to develop new interventions to deal with adverse reactions after medication.

The main contributions of this study include the accurate classification of actual ADR data, as well as the GAN and SMOTE methods used in this process, in an effort to realize the feature enhancement and minority oversampling. We verify that the model combining PRR, feature enhancement (FS_GAN), SMOTE, and RF classification is optimal for CFDA's spontaneous reporting data, and gives the evaluation metrics suitable for imbalanced data set. This study also provides reference for medical experts on the risk evaluation and status switch of post-marketing drugs.

## 7. Conclusions

This paper proposes a model combining feature enhancement (FS_GAN) and SMOTE for drug risk evaluation in CFDA's spontaneous reporting data. Based on the comparison of three sets of models, the classification accuracy of the proposed model is nearly 98%. The results suggest that the combination of PRR, FS_GAN, SMOTE, and RF method is determined to be the optimal framework for class-imbalance problems in ADR data. At the same time, the effective features generated by GAN have a significant contribution to the classification performance. This means GAN can be used in more classification scenarios to obtain better results.

This model has the potential to be generalized to more drug regulatory agencies, because it can provide a convenient and reliable way for the ADR signal detection and drug classification. The results will serve as a strong basis for experts to evaluate potential risk of drugs and help them make more judgmatic decisions for the switch of drug status. In the future, it is necessary to pay attention to the adverse reactions caused by the mutual influence of multiple drugs, which will help to further explore the relationship between different ingredients and reduce the risk of medication.

## Figures and Tables

**Figure 1:** Flowchart of the proposed model.

**Figure 2:** Confusion matrices based on the test set.

**Figure 3:** Confusion matrices based on the actual ADR data.

**Figure 4:** ROC curves and AUC values based on the actual ADR data.

**Table 1:** Quantity information of drugs in data set.

Drug category	Label	Sample size	Percentage
Rx	0	887	84.72
OTC-A	1	113	10.79
OTC-B	2	47	4.49

**Table 2:** DPA two-by-two contingency table.

	Target ADRs	Other ADRs	Total
Target drugs	*A*	*B*	*A* + *B*
Other drugs	*C*	*D*	*C* + *D*
Total	*A* + *C*	*B* + *D*	*A* + *B* + *C* + *D*

**Table 3:** Classification in the confusion matrix.

	Positive	Negative
True	True positive (TP)	True negative (TN)
False	False positive (FP)	False negative (FN)

TP: the number of samples that predict the positive class as a positive class. TN: the number of samples that predict the negative class as a negative class. FP: the number of samples that predict a negative class as a positive class. FN: the number of samples that predict a positive class as a negative class.

**Table 4:** Evaluation metrics based on the test set.

Classifier	Label	Precision	Recall	F1	Accuracy (%)
Model 1 (RF)	0	0.85	0.99	0.92	
	1	0.50	0.03	0.06	84.44
	2	0.00	0.00	0.00	
	Macro-avg	0.45	0.34	0.32	
	Weighted-avg	0.78	0.84	0.78	

Model 2 (SMOTE + RF)	0	0.91	0.85	0.88	
	1	0.91	0.94	0.92	91.99
	2	0.94	0.97	0.96	
	Macro-avg	0.92	0.92	0.92	
	Weighted-avg	0.92	0.92	0.92	

Model 3 (FS_GAN + SMOTE + RF)	0	0.93	0.96	0.94	
	1	0.98	0.94	0.96	96.25
	2	0.98	0.98	0.98	
	Macro-avg	0.96	0.96	0.96	
	Weighted-avg	0.96	0.96	0.96	

**Table 5:** Evaluation metrics based on the actual ADR data.

Classifier	Label	Precision	Recall	F1	Accuracy (%)
Model 1 (RF)	0	0.89	0.99	0.94	
	1	0.80	0.36	0.50	88.63
	2	0.72	0.28	0.40	
	Macro-avg	0.81	0.54	0.61	
	Weighted-avg	0.88	0.89	0.87	

Model 2 (SMOTE + RF)	0	0.98	0.95	0.97	
	1	0.80	0.90	0.85	94.65
	2	0.72	0.94	0.81	
	Macro-avg	0.83	0.93	0.88	
	Weighted-avg	0.95	0.95	0.95	

Model 3 (FS_GAN + SMOTE + RF)	0	0.99	0.99	0.99	
	1	0.92	0.93	0.93	97.90
	2	0.96	0.94	0.95	
	Macro-avg	0.96	0.95	0.95	
	Weighted-avg	0.98	0.98	0.98	

## Data Availability

All ADR spontaneous reporting data in this study are licensed by the CFDA. The data sets are not publicly available due to the policy of confidentiality of the CFDA but are available from the corresponding author on reasonable request and with permission of the CFDA.
